This article has been retracted.

# Progressive Familial Intrahepatic Cholestasis Type 2 in an Infant: Diagnostic Challenges and Multidisciplinary Management

**DOI:** 10.7759/cureus.76355

**Published:** 2024-12-25

**Authors:** Najeeb Ullah, Somaan Anthony, Arzoo Siddiqi, Nimra Akram, Bismil Afghan

**Affiliations:** 1 Internal Medicine, Rehman Medical Institute, Peshawar, PAK; 2 Internal Medicine, Lady Reading Hospital, Peshawar, PAK; 3 Internal Medicine, Dow University of Health Sciences, Karachi, PAK; 4 Internal Medicine, Jinnah Sindh Medical University, Karachi, PAK; 5 Internal Medicine, Nishtar Medical University, Multan, PAK

**Keywords:** abcb11 mutation, cholestasis, liver transplantation, pediatric liver disease, pfic2, progressive familial intrahepatic cholestasis

## Abstract

Progressive familial intrahepatic cholestasis type 2 (PFIC2) is a rare genetic disorder characterized by severe intrahepatic cholestasis, which often manifests in infancy with progressive liver dysfunction. We present the case of a 3-month-old infant with a one-month history of jaundice, vomiting, and bloody stools, presenting a unique set of diagnostic challenges. Initial clinical and laboratory findings indicated significant liver dysfunction, prompting further imaging and genetic analysis. An abdominal ultrasound revealed hepatomegaly with a coarse liver texture, while a hepatobiliary iminodiacetic acid (HIDA) scan ruled out biliary atresia. Ultimately, genetic testing confirmed a mutation in the ABCB11 gene, diagnostic of PFIC2. Management included total parenteral nutrition to support growth, ursodeoxycholic acid to improve bile flow, and rifampicin to alleviate pruritus. Due to the severity of the disease, a liver transplant is planned as the definitive treatment following stabilization through supportive care. This case underscores the importance of a high index of suspicion, timely genetic testing, and a multidisciplinary approach in managing PFIC2 to optimize patient outcomes.

## Introduction

Progressive familial intrahepatic cholestasis (PFIC) is a rare group of autosomal recessive genetic disorders characterized by impaired bile flow (cholestasis) within the liver, leading to progressive liver disease, often starting in infancy or early childhood. PFIC is divided into three primary subtypes (PFIC1, PFIC2, and PFIC3), each caused by mutations in specific genes involved in bile transport. These mutations disrupt the mechanisms essential for bile secretion, resulting in cholestasis and liver damage over time [1]. PFIC is rare, with an estimated incidence of 1 in 50,000 to 1 in 100,000 live births [2]. As an autosomal recessive disorder, PFIC requires both parents to be carriers of a mutated gene for a child to inherit the condition.

PFIC typically presents within the first few months of life, with symptoms such as jaundice, pruritus, and growth impairment. The clinical presentation and severity of symptoms vary across PFIC subtypes, with PFIC2 often leading to more severe liver dysfunction early in life compared to other types. The disease progresses to end-stage liver disease in many cases, necessitating liver transplantation as the definitive treatment [3]. This case report aims to expand the clinical understanding of PFIC, specifically PFIC2, by providing a detailed account of its diagnosis, management, and outcomes. By documenting the clinical presentation, diagnostic challenges, and therapeutic strategies, this report seeks to assist clinicians and researchers in improving diagnostic accuracy, optimizing patient outcomes, and advancing therapeutic options for PFIC.

## Case presentation

A 3-month-old full-term infant presented to the hospital with a one-month history of jaundice, characterized by yellow discoloration of the eyes and skin. The mother noted that the yellowing of the skin developed suddenly and progressively worsened, with the eyes becoming markedly pale. Along with the jaundice, the infant experienced vomiting after breastfeeding, which occurred immediately following feeds. This contributed to significant nutritional challenges, resulting in weight loss and poor growth. Notably, the vomiting was not associated with fever or facial flushing.

In addition to the jaundice and vomiting, the mother reported the infant passing blood-streaked stools for the past 15 days. Initially, the blood was bright red, but it later turned dark and blackish. The amount of blood was minimal and easily flushed away, with no associated fever. The infant's delivery was uncomplicated, achieved through spontaneous vaginal delivery (SVD), and feeding consisted of a combination of breastfeeding and formula supplementation. The family history was notable for similar symptoms in a previous generation, with a known history of consanguinity, as the infant's parents were cousins.

On physical examination, the infant appeared emaciated and lethargic, with significant jaundice and pallor. The sclerae were markedly yellow, consistent with severe hyperbilirubinemia. Abdominal examination revealed hepatomegaly, with the liver palpable two fingers below the right subcostal margin, while the spleen was non-palpable. The infant exhibited reduced activity levels and was generally inactive, although all neonatal reflexes were intact. Vital signs were within normal limits for age, with no fever or signs of acute distress.

Based on the clinical presentation, the primary differential diagnoses included progressive PFIC and biliary atresia. Both conditions share overlapping features, such as jaundice, vomiting, hepatomegaly, and poor nutritional status. PFIC was suspected due to the progressive nature of the jaundice and family history of a similar illness, especially considering the consanguineous marriage of the parents. Biliary atresia remained a strong consideration, given the significant jaundice and liver enlargement. To further refine the diagnosis and guide management, a series of targeted investigations was initiated. Baseline investigations (Table 1) revealed significant liver dysfunction, indicated by marked hyperbilirubinemia, elevated liver enzymes, and notable hematological abnormalities.

**Table 1:** Key laboratory findings indicative of hepatic dysfunction. INR: international normalized ratio, ALT: alanine transaminase, AST: aspartate aminotransferase, ALP: alkaline phosphatase.

Investigation	Result	Reference range
Prothrombin time	14 seconds	Up to 13 seconds
INR	1.17	0.9-1.3
Hemoglobin	5.80 g/dL	13-18 g/dL
Platelets	30 x 10^9^/L	150-400 x 10^9^/L
Total bilirubin	10.6 mg/dL	0.3-1.2 mg/dL
Direct bilirubin	6.68 mg/dL	<0.3 mg/dL
ALT	114 U/L	Up to 40 U/L
AST	228 U/L	Up to 40 U/L
ALP	566 U/L	40-120 U/L
Serum creatinine	0.19 mg/dL	0.5-0.9 mg/dL
Bilirubin (urine)	30 umoL/L	Negative
Protein (urine)	Trace	<150 mg/dL

An ultrasound (US) of the abdomen and pelvis revealed hepatomegaly with a coarse liver texture and a partially filled gallbladder. These findings suggested liver dysfunction but were nonspecific for biliary atresia. To further evaluate the condition, a hepatobiliary iminodiacetic acid (HIDA) scan was conducted, which showed normal bile flow, ruling out biliary atresia as the primary diagnosis. Given the clinical presentation and imaging findings, PFIC was strongly suspected. Genetic testing was subsequently performed, which confirmed a mutation in the ABCB11 gene located on chromosome 2q24, establishing a diagnosis of PFIC2. Figure 1 shows the liver US image.

**Figure 1:** Ultrasound of the liver, oblique scan. There is an increase in hepatic volume and a slight decrease in echostructure, while the walls of the portal branches appear brighter.

Upon diagnosis, the infant was started on symptomatic and supportive management. To address malnutrition and prevent further weight loss, total parenteral nutrition (TPN) was initiated, ensuring that the infant received adequate nutrients to support growth. Low-dose antibiotics were administered to prevent secondary infections, which were a concern due to the infant's compromised liver function and reduced immunity. Due to the infant’s severe anemia and thrombocytopenia, blood transfusions were administered to maintain safe levels of hemoglobin, red cell counts, and platelets. This intervention was essential to manage the risk of bleeding, especially in the context of portal hypertension.

In preparation for a liver transplant, which is considered the gold-standard treatment for PFIC, the care team focused on stabilizing the infant's condition. Nasobiliary drainage was planned to reduce hepatic stress and alleviate jaundice symptoms. Additionally, medications such as ursodeoxycholic acid were introduced to improve bile flow, and rifampicin was prescribed to help manage pruritus associated with cholestasis. The infant also exhibited signs of portal hypertension, as evidenced by bloody stools, so vasopressors were administered to help stabilize blood pressure and manage complications related to elevated portal pressures.

During the follow-up period, the infant’s weight and nutritional status gradually improved due to parenteral nutrition and controlled feeding regimens. Liver function tests were closely monitored, showing only slight improvements, confirming the need for liver transplantation as a definitive treatment. The planned liver transplant procedure will provide the infant with a functional liver, restoring normal bile transport and addressing the underlying cause of PFIC2.

## Discussion

This case of a 3-month-old infant presenting with jaundice, vomiting, and bloody stools underscores the unique challenges in diagnosing and managing progressive PFIC2, a rare genetic disorder. The early onset of severe jaundice and gastrointestinal bleeding highlights the importance of prompt clinical evaluation in neonates with persistent cholestasis. This case was further complicated by overlapping features with other conditions, such as biliary atresia, necessitating a combination of imaging, biochemical tests, and genetic analysis to achieve a definitive diagnosis. The multidisciplinary approach, involving pediatric hepatologists, geneticists, nutritionists, and transplant surgeons, played a pivotal role in stabilizing the infant, addressing nutritional deficits, and planning for liver transplantation. This case emphasizes the importance of early recognition, comprehensive diagnostic strategies, and collaborative care in optimizing outcomes for infants with complex hepatic disorders.

The clinical presentation of this case, marked by jaundice, vomiting, and bloody stools, aligns with previously reported cases of PFIC2, where early-onset jaundice and progressive liver dysfunction are hallmark features [4]. However, the presence of bloody stools in this infant is less commonly reported in PFIC2, likely stemming from advanced complications such as portal hypertension and coagulopathy, as supported by studies highlighting gastrointestinal bleeding in advanced stages of the disease [5]. The diagnostic challenges faced in this case mirror those documented in the literature, particularly the difficulty in differentiating PFIC2 from biliary atresia due to overlapping symptoms like persistent jaundice and hepatomegaly. Genetic testing, which confirmed a mutation in the ABCB11 gene encoding the bile salt export pump (BSEP), proved instrumental in establishing a definitive diagnosis, consistent with its role as the diagnostic gold standard in similar studies [6]. Management strategies in this case emphasized supportive care, including parenteral nutrition and pharmacological interventions such as ursodeoxycholic acid and rifampicin, paralleling established therapeutic approaches [7]. However, the planned liver transplantation underscores the necessity of surgical intervention in severe cases, reflecting the findings of previous studies that highlight transplantation as the definitive treatment for PFIC2, especially in cases unresponsive to medical therapy.

The diagnosis of PFIC2 presents significant challenges due to its clinical overlap with other cholestatic disorders, such as biliary atresia, which also manifests with persistent jaundice, hepatomegaly, and failure to thrive in infants [8]. In this case, the differentiation was particularly complex, as initial imaging findings, including hepatomegaly with a coarse liver texture, were nonspecific. The use of a hepatobiliary iminodiacetic acid (HIDA) scan to rule out biliary atresia, combined with confirmatory genetic testing that identified a mutation in the ABCB11 gene, exemplifies the critical role of advanced diagnostic tools in establishing a definitive diagnosis. The multidisciplinary approach was equally pivotal in the management of this infant, involving pediatric hepatologists, geneticists, nutritionists, and transplant surgeons. This collaboration ensured comprehensive care, addressing nutritional deficits through parenteral nutrition, managing symptoms with targeted pharmacological interventions, and preparing for a liver transplant. By leveraging the expertise of a diverse team, this case highlights the importance of an integrated approach to optimize outcomes and provide a clear path toward definitive treatment in complex genetic disorders like PFIC2.

This case underscores several critical lessons for the early diagnosis and management of PFIC2, particularly the importance of promptly recognizing symptoms such as persistent jaundice and nutritional deficits to prevent severe complications like portal hypertension and coagulopathy [9]. Early intervention with supportive care, including parenteral nutrition and pharmacological agents like ursodeoxycholic acid, played a vital role in stabilizing the infant. The case also highlights the importance of genetic counseling, especially in consanguineous families, to identify carriers and provide preemptive guidance for future pregnancies. Looking ahead, emerging therapeutic options, including gene therapy and bile salt export pump modulators, offer hope for addressing the genetic defect in PFIC2 [10]. Additionally, targeted drugs aimed at reducing bile acid toxicity and improving hepatocyte function are under investigation, potentially providing alternatives to invasive treatments like liver transplantation and paving the way for more personalized approaches to managing this rare but severe disorder.

Current diagnostic and treatment modalities for PFIC2 remain limited, with challenges in early detection due to overlapping symptoms with other cholestatic disorders and reliance on genetic testing, which may not be readily accessible in resource-limited settings. Treatment primarily focuses on supportive care and liver transplantation, the latter being invasive and not universally available. Future research should aim to develop noninvasive diagnostic tools, enhance access to genetic testing, and explore early intervention strategies. Additionally, advancements in gene therapy, bile salt export pump modulators, and other targeted therapies offer promise as less invasive and more accessible alternatives to liver transplantation, addressing a significant gap in the management of PFIC2.

## Conclusions

This case of a 3-month-old infant with progressive PFIC2 highlights the importance of early recognition and multidisciplinary management of this rare yet severe genetic disorder. The clinical presentation, characterized by jaundice, vomiting, and signs of portal hypertension, along with confirmatory genetic testing, underscores the need for high clinical suspicion in infants presenting with persistent cholestasis. The planned liver transplantation, following supportive measures and pharmacologic interventions, offers the best prognosis as the definitive treatment for this infant. This case emphasizes that timely diagnosis, comprehensive supportive care, and genetic counseling are vital for optimizing outcomes, ultimately enhancing survival and quality of life for infants affected by PFIC2.
